The article "Phytoremediation of nickel by quinoa: Morphological and physiological response" was retracted in 2022. Reasons: compromised peer review; a conflict of interest; concerns about the authorship.

# Phytoremediation of nickel by quinoa: Morphological and physiological response

**DOI:** 10.1371/journal.pone.0262309

**Published:** 2022-01-13

**Authors:** Muhammad Haseeb, Shahid Iqbal, Muhammad Bilal Hafeez, Muhammad Sohail Saddiq, Noreen Zahra, Ali Raza, Muhammad Usman lbrahim, Javaid Iqbal, Muhammad Kamran, Qasim Ali, Talha Javed, Hayssam M. Ali, Manzer H. Siddiqui

**Affiliations:** 1 Department of Agronomy, University of Agriculture, Faisalabad, Pakistan; 2 Department of Agronomy, Muhammad Nawaz Shareef, University of Agriculture, Multan, Pakistan; 3 Department of Agronomy, Ghazi University, Dera Ghazi Khan, Pakistan; 4 Department of Botany, University of Agriculture, Faisalabad, Pakistan; 5 Fujian Provincial Key Laboratory of Crop Molecular and Cell Biology, Oil Crops Research Institute, Centre of Legume Crop Genetics and Systems Biology/College of Agriculture, Fujian Agriculture and Forestry University, Fuzhou, China; 6 Institute of Food and Agriculture Sciences, University of Florida, Gainesville, FL, United States of America; 7 College of Agriculture, Fujian Agriculture and Forestry University, Fuzhou, China; 8 Department of Botany and Microbiology, College of Science, King Saud University, Riyadh, Saudi Arabia; The University of Haripur, PAKISTAN

## Abstract

The amount of soil contaminated with heavy metal increases due to urbanization, industrialization, and anthropogenic activities. Quinoa is considered a useful candidate in the remediation of such soil. In this pot experiment, the phytoextraction capacity of quinoa lines (A1, A2, A7, and A9) against different nickel (Ni) concentrations (0, 50, and 100 mg kg^-1^) were investigated. Required Ni concentrations were developed in polythene bags filled with sandy loam soil using nickel nitrate salt prior to two months of sowing and kept sealed up to sowing. Results showed that translocation of Ni increased from roots to shoots with an increase in soil Ni concentration in all lines. A2 line accumulated high Ni in leaf compared to the root as depicted by translocation factor 3.09 and 3.21 when grown at soil having 50 and 100 Ni mg kg^-1^, respectively. While, in the case of root, A7 accumulated high Ni followed by A9, A1, and A2, respectively. There was a 5–7% increased seed yield by 50 mg kg^-1^ Ni in all except A1 compared to control. However, growth and yield declined with a further increase in Ni level. The maximum reduction in yield was noticed in A9, which was strongly linked with poor physiological performance, e.g., chlorophyll a, b, and phenolic contents. Ni concentrations in the seed of all lines were within the permissible value set (67 ppm) by FAO/WHO. The result of the present study suggests that quinoa is a better accumulator of Ni. This species can provide the scope of decontamination of heavy metal polluted soil. The screened line can be used for future quinoa breeding programs for bioremediation and phytoextraction purpose.

The article "Phytoremediation of nickel by quinoa: Morphological and physiological response" was retracted in 2022. Reasons: compromised peer review; a conflict of interest; concerns about the authorship.

## 1. Introduction

Worldwide, dealing with heavy metals toxicity is a major challenge for agricultural scientists because they are in soil environment have become a leading health concern, especially for plants, humans, and animals [1–3]. Due to anthropogenic sources, heavy metals toxicity is increasing in the soil. Among different metals, nickel (Ni) contamination is one of the leading heavy metals that comes from the discharge of effluents from industries, i.e., Ni steel and iron alloys [4], cadmium batteries [5], electroplating [6], and also by the application of pesticide and municipal wastes [7]. Besides these facts, excessive Ni in the land has become a devastating threat to crops’ growth, development, and productivity [8]. Ni toxicity reduced the intake of CO_2_, declined photosynthesis, chlorophyll contents, and relative water [9], and impaired cell division and elongation [10]. Consequently, the initiation of oxidative damage annoys the balance between antioxidants and reactive oxygen species (ROS) [11], damaging the nucleic acids, proteins, and organelles’ membranes [12].

The management of heavy metals has become crucial to minimize the arising adverse effects on soil, plant, and the environment [2, 13, 14]. Plants have developed metal tolerance mechanisms, chelation, and compartmentalization to maintain trace element homeostasis [15–17]. Therefore, different techniques have been employed in the successful removal of Ni from the soil, such as excavation, electrokinetic, incineration, soil washing (complex, costly, and damage soil quality and fertility), bioremediation, and phytoremediation (ecofriendly and not disturbing the soil fertility and biodiversity) [18–21]. Among them, the growing of hyperaccumulating plant species (phytoremediation) is a good option to cope with elevated Ni in their shoots without expressing toxicity symptoms, and also developed an enzymatic and non-enzymatic antioxidant mechanism which can alleviate oxidative damage to organelles by scavenging ROS species, thereby resulted in higher grain yield [22, 23]. This approach not only removes heavy metals from the soil but also cleans the environment from other pollutants. These heavy metals need to be removed from the soil for agro-ecological sustainability and human benefits. The use of the plant for remediation of heavy metal or phytoextraction is an exciting approach nowadays [24–26]. Phytoextraction requires translocation of heavy metal from contamination surface to harvest stable part [27].

The article "Phytoremediation of nickel by quinoa: Morphological and physiological response" was retracted in 2022. Reasons: compromised peer review; a conflict of interest; concerns about the authorship.

*Chenopodium spp*. has the genetic ability to accumulate large quantities of heavy metal in leaf tissue. *C*. *quinoa* is a better accumulator of Cr, Cd, and Ni and detoxifies contaminated soils [24, 25]. Quinoa has a deep taproot and fibrous root system that allows quinoa plants to access nutrient and soil water unavailable to other plants. These growing characteristics may enhance the uptake efficiency for trace elements [28]. Quinoa is a hyperaccumulator of Pb, Cd, and nickel in the early stages of growth and removes more metals from the soil when grown to maturity [29]. It has gained attention globally due to its high nutritional and health benefits and the ability to grow under contaminated environments [30, 31]. Pakistan is an underdeveloped country, not focusing on the industrial waste containing heavy metals affecting the agricultural soil. Therefore, it is important to determine the morphological and physiological responses, phytoextraction ability, and yield potential of quinoa under Ni-contaminated soils.

## 2. Materials and methods

### 2.1. Plant material and Ni imposition

A pot trial was executed during winter 2014–15 in a wirehouse (natural environment), Department of Agronomy, University of Agriculture Faisalabad (UAF), Pakistan. Quinoa lines were taken from Alternate Crops Lab, Department of Agronomy, UAF, and the details of lines (A1, A2, A7, and A9) are given in Table 1. Local codes were used to quote respective lines during the study. In order to remove extraneous matter, collected soil samples were air-dried and sieved using a 2 mm sieve and processed to determine physio-chemical characteristics as presented in Table 2. The experiment was carried out in plastic pots (18 cm height and 20 cm base) with 5 kg of the sieved soil. As per the metal concentration of global soils, 0, 50, and 100 mg kg^-1^ concentrations of Ni were selected [32, 33]. At the same time, 50 and 100 mg kg^-1^ aqueous solution of Ni was prepared according to respective treatments. The source was analytical grade nickel nitrate Ni(NO_3_)_2_ (Sigma-Aldrich), applied to corresponding pots with three replicates. After two months of Ni treatments, seeds of quinoa lines were sown in pots. Fifteen seeds of each quinoa line were sown in each pot. Pots were placed in wire house under ambient light and temperature. The recommended dose of fertilizers (N:P:K @75:60:60 kg ha^-1^) as urea, diammonium phosphate, and sulfate of potash were applied to each pot. The experiment was conducted using a completely randomized design (CRD) with a factorial arrangement. After emergence, five plants per pot were maintained, and irrigations were applied according to the water requirement of plants. 250 ml distal water per plot was applied daily, and pots were non-leachable.

The article "Phytoremediation of nickel by quinoa: Morphological and physiological response" was retracted in 2022. Reasons: compromised peer review; a conflict of interest; concerns about the authorship.

**Table 1:** Detail of quinoa lines used in the current study.

Code*	G. Line **	Origin	Plant name
P1 596293	A1	Colorado, USA	Colorado 407D
Ames 13730	A2	New Mexico, USA	IESP
Ames 13737	A7	New Mexico, USA	2WANT
P1 634919	A9	Chile	Pichaman

(* as per the germplasm database **coding of lines made for local identification).

**Source:** The main source was USDA since 2008.

**Table 2:** Physico-chemical analysis of pot soil used in the current study.

Determination	Unit	Value
pH	---	7.6
EC	dS m^-1^	0.93
Nitrogen	mg kg^-1^	0.043
Phosphorus	mg kg^-1^	13.11
Potassium	mg kg^-1^	87
Cadmium	^---^	0.36
Chromium		2.3
Lead		0.07
Nickel		0.44
Organic Matter		0.88
Textural Class		Sandy loam

### 2.2. Growth parameters

Eighty days after sowing, plants from each pot were carefully uprooted and separated into shoots and roots by which root is not damaged. Shoot and root length (cm) were measured using a foot ruler. For root and shoot fresh weights (g), plants were washed with a gentle stream of water. After that, their weights were noted with an analytical balance. Shoot and root samples were oven-dried at 70°C for 72 h, then dry shoot and root weights (g) were noted.

### 2.3. Nickel determination

The determination of Ni was done according to the method of Wolf [34], by which 5 mL of HNO_3_ was taken in each digestion flask containing 0.1 g of dried sample of leaf, root, stem, and seeds (0.1 g). Then incubated the same samples were overnight at room temperature and heated on a hot plate at 250°C until fumes were formed. After that, heating continued again for 30 min and added 1 mL of HNO_3_ in each flask on cooling and placed back on a hot plate for heating. The same process repeated as described above until the material became clear and colorless. Then, made the volume upto 50 mL using distilled water. The extract was filtered to determine readings using an Atomic Absorption Spectrophotometer (Hitachi Polarized Zeeman AAS, Z8200, Japan) following the procedure as described in [35].

### 2.4. Physiological attributes

Determinations of Chlorophyll a, b, and carotenoids were measured using the procedure of Arnon [36], and Davis and Goodwin [37], respectively. Briefly, leave samples (0.5 g) were collected at 80 DAS (panical emergence stage) and homogenized in 80% acetone by pestle and mortar under a dark chamber. Then, filtered and made the volume upto 10 mL. Further, 663, 645, and 480 nm UV-V is spectrophotometer (Dynamica Co., UK; Halo DB-20/DB 20S) wavelength was used to determine chlorophyll a, b carotenoids, respectively. The following formula was used for the determination of chlorophyll and carotenoids:

Chlorophyll a (mg/g fresh wt.) = (1.27 (OD663)-2.69(OD645) ×V/1000×W

Chlorophyll b (mg/g fresh wt.) = (22.9 (OD645)-4.68(OD663) ×V/1000×W

Carotenoids (mg/g fresh wt.) = (OD480+0.114(OD663)-0.638 (OD645)/2500) × 1000

For the determination of phenolics, according to Julkunen-Tiitto [38], 80% acetone was used to get an extract of 0.5 g leave sample. Then, the same extract was centrifuged at 12,000 rpm for 5 min, and 100 μL of the extract was mixed in Folin-Ciocalteu’s phenol reagent (0.5 mL), and 2.5 mL of 20% Na_2_CO_3_. After that, distilled water was used to make volume upto 5 mL and vortexed for recording absorbance at 750 nm.

The article "Phytoremediation of nickel by quinoa: Morphological and physiological response" was retracted in 2022. Reasons: compromised peer review; a conflict of interest; concerns about the authorship.

### 2.5. Translocation factor (TF)

TF was calculated following the formula of Liu et al. [39].

TF = Metal concentration in shoot (mg/kg)/Metal concentration in root (mg/kg)

### 2.6. Yield and yield-related attributes

Before harvesting, the number of panicles was counted from each pot, and panicle length (cm) was recorded by using a foot ruler. Following the method as described by Jacobsen and Stølen [40], harvested panicles were dried at 25‒30°C using filter paper, and threshing was done manually after ten days. Then, the dry weight and total crop biomass were calculated after sun-drying the samples for a week. Electric balance was used to calculate thousand seed weights.

### 2.7. Statistical analysis

A two-way ANOVA analysis was conducted to analyze the data for a completely randomized design (CRD) that replicated thrice under factorial arrangement with the help of statistical software “Statistics” (ver. 8.1, Tallahassee, FL, USA). R-software (corrplot package) was used to draw correlations among different response variables.

## 3. Results

### 3.1. Effect of Ni on growth parameters

All quinoa lines differed significantly for shoot and root length under control and Ni stress conditions. Under maximum Ni application (100 mg kg^-1^), A1 and A2, unlike other lines, showed a maximum increment in shoot length (2.4 and 1.6%), respectively (Fig 1A). While both these lines showed an increase in root length (6.45 and 2.43%) at a lower Ni dose (50 mg kg^-1^) as compared to control (Fig 1B).

**Fig 1:** Influence of different Ni concentrations on growth parameters (a) shoot length; (b) root length; (c) shoot fresh weight; (d) shoot dry weight; (e) root fresh weight; and (f) root dry weight, of four quinoa lines. Error bars denote the standard error of three replications. Bars with the same letters do not differ significantly at p ≤ 0.05.

For shoot dry weight, A7 and A9 exhibited no significant increase between control and 100 mg kg^-1^ Ni treatment but A1 and A2 lines displayed (2.76 and 11.13%) at 50 mg kg^-1^ and (0.85 and 7.54%) increment at 100 mg kg^-1^ Ni application, respectively (Fig 1D). Quinoa A2, unlike other lines, manifested a substantial decline of root dry weight at 50 and 100 mg kg^-1^ Ni compared to control (Fig 1F).

The article "Phytoremediation of nickel by quinoa: Morphological and physiological response" was retracted in 2022. Reasons: compromised peer review; a conflict of interest; concerns about the authorship.

### 3.2. Effect of Ni on physiological parameters

The photosynthetic pigments of Ni-treated lines were gradually decreased. For instance, compared to control, the maximum reduction of chl *a* recorded 34, 21.36, 18.86, and 7.86% in A9, A7, A1, and A2 lines, respectively. On the other hand, chl *b* content decreased 19.53, 16.51, 12.63, and 8.51 in A7, A1, A2, and A9 lines at 100 mg kg^-1^ Ni application, respectively (Fig 2A and 2B). A minor reduction was observed in carotenoid contents in all lines except A2, in which the values did not significantly reduce (Fig 2C). Compared to other lines, the A2 line showed a higher aptitude to accumulate (57.7%) phenolic at 100 mg kg-1Ni exposure (Fig 2D).

**Fig 2:** Influence of Ni concentrations on (a) Chl a; (b) Chl b; (c) carotenoids; and (d) soluble phenolic. Error bars denote the standard error of three replications. Bars with the same letters do not differ significantly at p ≤ 0.05.

### 3.3. Nickel accumulation and translocation

This study was determined in terms of the variable phytoextraction potential of four quinoa lines regarding Ni accumulation. The determination made for Ni contents in (leaf, stem, root, and seed) indicated a significant (P<0.01) difference among treatments in quinoa grown in Ni-contaminated pots.

Analysis of leaf Ni concentration at all three harvests (multiple leaves stage, panicle emergence stage, and before harvesting) showed a significant increase in Ni concentration in all quinoa lines with an increase in duration and Ni doses. The pattern is followed by quinoa lines (A2>A1>A7>A9) in all three harvests for leaf Ni. At the 2^nd^ harvest (panicle emergence stage), Ni concentration was (10494.7 and 15610.5%) increased in A2 at 50 and 100 mg kg^-1,^ respectively, in comparison to control (Fig 3A).

**Fig 3:** Nickel concentration in plant parts (a) leaf; (b) stem; and (c) root, and (d) translocation factor. Error bars denote the standard error of three replications. Bars with the same letters do not differ significantly at p ≤ 0.05.

For all quinoa lines, a significant increase in stem Ni concentration was observed when soil Ni was increased from 50 mg kg^-1^ to 100 mg kg^-1^. In the A9 line, the Ni concentration in the stem did not exceed (3.26 mg kg^-1^) with 100 mg kg^-1^ Ni application. However, A1 succeeded in absorbing (3.03 and 5.1 mg kg^-1^) nickel with (50 and 100 mg kg^-1^) Ni dose respectively before harvest (Fig 3B).

The article "Phytoremediation of nickel by quinoa: Morphological and physiological response" was retracted in 2022. Reasons: compromised peer review; a conflict of interest; concerns about the authorship.

An increase in Ni doses enhanced the root nickel absorbance of quinoa lines, but maximum increment (3125 and 4950%) with use of (50 and 100 mg kg^-1^) was observed in A7 compared to control. Contrarily, the lowest root Ni concentration was noted in A2 as compared to other lines. Translocation factor (TF) is used as a tool to access the phytoextraction potential of quinoa lines to remediate the Ni-contaminated soil. An increasing trend was noted in all lines with increasing application of Ni level in an external environment (Fig 3C). The value of TF was recorded maximum in A2 at all three harvests as compared to other lines. Nickel application enhanced translocation value from 0.60 (control) up to 3.09 and 3.21 at (50 and 100 mg kg^-1^) Ni doses, respectively, at panicle emergence stage (80 days after sowing) in comparison to data of other two harvests (40 and 120 days after sowing) (Fig 3D).

The Ni translocation from shoot to seed was observed in all quinoa lines. Maximum seed Ni was found in A7 (1036.5 and 1729.2%) with an application of (50 and 100 mg kg^-1^) Ni, respectively, compared to control. The trend of quinoa lines regarding Ni storage in seed was A7>A2>A9>A1 (Fig 4E).

**Fig 4:** Influence of Ni concentrations on (a) panicle length; (b) the number of panicle; (c) biological yield; (d) seed yield; (e) 1000-seed weight; and (f) seed nickel of four quinoa lines. Error bars denote the standard error of three replications. Bars with the same letters do not differ significantly at p ≤ 0.05. Add the meaning of different lower case letters.

### 3.4. Effect of Ni on yield-related parameters

Applied Ni slightly increased panicle length (3.74 and 3.44%) in A1 and A2 lines respectively at 50 mg kg^-1,^ whereas high application (100 mg kg^-1^) improved panicle length (3.44%) in the A2 line. The data indicated that Ni application improved (6.45 and 3.22%) panicles number in A2 at 50 and 100 mg kg^-1^ nickel, respectively. In the A2 line, the biological and seed yield increased at 50 mg kg^-1^, then a slight reduction was observed at (100 mg kg^-1^) Ni, while A7 and A9 displayed a decline in these character at both (50 and 100 mg kg^-1^) Ni levels (Fig 4).

### 3.5. Correlation analysis

A Pearson’s correlation analysis was performed between diverse studied parameters of quinoa under different Ni concentrations (Fig 5). Under 0 mg kg^-1^ Ni level, LNi was negatively correlated with SL and RL. Further, Niseed, BY, SY SNi were negatively correlated with LNi. At the same time, all other parameters were positively correlated with each other (Fig 5A). In response to 50 mg kg^-1^ Ni, RNi was negatively correlated with RL, LNi, and SNi. Likewise, Niseed, BY, and SY were negatively correlated with RNi; however, all other parameters were positively correlated (Fig 5B). In response to 100 mg kg^-1^ Ni, RNi and SNi were negatively correlated with SL, RL, and LNi. Moreover, Niseed, BY and SY were also negatively correlated with SNi and RNi; nonetheless, other parameters were positively correlated (Fig 5C). Overall, the correlation analysis revealed a strong correlation between SY, BY, Niseed, LNi, RL, and SL induced by different Ni concentrations.

The article "Phytoremediation of nickel by quinoa: Morphological and physiological response" was retracted in 2022. Reasons: compromised peer review; a conflict of interest; concerns about the authorship.

**Fig 5:** Pearsons correlation analysis between different studies parameters under (a) 0 mg kg-1 Ni, (b) 50 mg kg-1 Ni, and (c) 100 mg kg-1 Ni concentrations. Correlation with color shows the strength of the connection of all experimental parameters. Blue and red colors indicate positive and negative correlation, respectively. Abbreviations: shoot length (SL), root length (RL), leaf Ni contents (LNi), stem Ni contents (SNi), root Ni contents (RNi), Ni in seed (Niseed), biological yield (BY), and seed yield (SY).

## 4. Discussion

The use of the plant, e.g., quinoa as phytoextraction, is an exciting approach nowadays [24–26]. The present study indicated that four quinoa lines showed differential responses regarding Ni accumulation. Shoot and root length and fresh and dry biomass of A1 and A2 lines were slightly high at 50 mg kg^-1^ Ni treatment. For most of these parameters, A1 and A2 displayed better growth at 50 and 100 mg kg^-1^ Ni than other quinoa lines.

However, quinoa lines A7 and A9 reduced their growth with increased Ni concentrations and exposure time. It suggests that the A1 and A2 entail some specific mechanisms to endure the Ni toxicity. Quinoa showed growth promotion at a low amount of metals [41]. Since Ni is an essential micronutrient for plants [42], the low amount is very useful and can improve plant growth [43]. It is well known that Ni is an essential metal for plants metabolism as it plays a key role in enzymes synthesis [44].

Chenopodium species have been documented to show differences for accumulating several heavy metals in the aerial parts [24]. For instance, Al-Whaibi, Siddiqui [45] reported that the growth of wheat was decreased with Ni application. In response to Ni contamination, wheat plants showed pitiable root growth and leaf blade reduction that leads to growth inhibition in wheat [46]. Furthermore, Gabbrielli, Pandolfini [47] reported that growth reduction under Ni treatment is generally related to loss of cellular turgor resulting in inhibit mitotic activity and delay of cell elongation.

Nickel can compete with other metals in absorbance due to similar characteristics of nickel with other metals. Therefore, Ni at high concentration inhibits the translocation of other essential metal ions leading to deficiency of other metals in plants [48]. Subsequently, this is the first step in plants to show toxicity and ultimately affect physiological processes [43]. As Ni impedes the translocation of Fe and Mg via competition, this could result in the delay of germination, growth, and yield reduction [49, 50]. Heavy metal toxicity interrupts the biochemical and physiological traits. Production of ROS is the first response to heavy toxicity. Overproduction of ROS results in oxidative stress. However, the secondary sequence of heavy metal stress is a disturbance in the electron transport chain, nutrient homeostasis, and antioxidant system [11, 51].

The article "Phytoremediation of nickel by quinoa: Morphological and physiological response" was retracted in 2022. Reasons: compromised peer review; a conflict of interest; concerns about the authorship.

Heavy metal toxicity lowered the nitrogen, protein content, carotenes, chlorophyll content, and hill reaction [15, 51] as reported in this study that chlorophyll contents were reduced gradually with an increase in Ni concentration in four quinoa lines (Fig 2A and 2D). Haseeb and Maqbool [52] documented the reduction of photosynthetic pigments in sunflower under stress conditions at the reproductive stage. With other heavy metals, Ni is destructive for plant photosynthetic mechanisms and disrupts the electron transport system. Previous reports indicated that Ni mainly accumulates in lamella regions of PSII and hampers photosynthesis [49]. Heavy metal toxicity lowered the nitrogen, protein content, carotenes, chlorophyll content, and hill reaction [24]. A high concentration of heavy metal, e.g., Pb, reduced the growth and photosynthetic pigment. Lead concentration adversely affects the chloroplast structure, which results in reduced enzyme activity, reduced CO_2_ fixation, and photosynthetic efficiency [24, 25].

In addition, carotenoid has a key role as accessory light-harvesting pigments; accumulation of carotenoid content is also advantageous in annulling oxidative damage caused by heavy metals [53]. It is plausible that greater carotenoid content is also beneficial in abolishing oxidative damage caused by heavy metals and thus protects photosynthetic pigments in the photosystems [53].

Nickel toxicity leads substantial increase in hydroxyl radicles, hydrogen peroxide, and nitric oxide. In response to oxidative stress, plants show induction of enzymatic and non-enzymatic antioxidant defense [54]. Among the non-enzymatic defense, phenolic compounds are important [55, 56]. In this study, data were recorded on the accumulation of soluble phenolic in the control and Ni-treated plants. Reports showed that soluble phenolic is accumulated under Ni toxicity [57]. Metal accumulation leads to an increase in phenolic concentration and maintained membrane integrity [57]. Metal binds with the hydroxyl and carboxyl groups of phenolic and have been identified as metal chelators and thus have a role in minimizing the deleterious effects of metal toxicity [58].

The article "Phytoremediation of nickel by quinoa: Morphological and physiological response" was retracted in 2022. Reasons: compromised peer review; a conflict of interest; concerns about the authorship.

The total amount of Ni absorbed by shoot is considered an important factor in evaluating a plant’s phytoextraction potential. The current study results revealed that All lines accumulated Ni, but A1 and A2 showed more intend to store it in leaf rather than roots without showing any adverse effect in the plant. Heavy metals are absorbed by roots, induce leaf chlorosis, inhibit root growth, and cause the deficiency of essential elements in most plants [15]. Symptom of heavy metal toxicity appeared on young leaves with the formation of dark green ribs. Under the toxicity, leave becomes chlorotic and turns white. Heavy metal toxicity reduced the germination and seedling growth traits, e.g., rice [15] in wheat [59]. Accumulation of a high nickel concentration caused the necrosis and chlorosis in the leaf, i.e., rice. Higher concentration of Ni has impaired membrane, disturbing lipid composition and nutrient homeostasis as Ni toxicity [15].

Nickel was very efficiently sequestered in the leaves of A2 without causing more adverse effects on photosynthetic pigments shows its better tolerance mechanism than other lines. [26] reported that quinoa has a deep taproot system that allows this plant to access soil water and nutrients. This characteristic may enhance the uptake efficiency for trace elements. Quinoa is a hyperaccumulator of Pb, Cd, and nickel in the early stages of growth and removes more metals from the soil when grown to maturity [29].

In the light of previous reports, a possible mechanism adopted by plants for efficient sequestration is the formation of complexes with ligands or compartmentalize into vacuole or cell wall. However, Ni peptide and Ni histidine complexes could also be responsible for Ni transport associated with citrate and malate [60].

Nickel is transported from roots to shoots and leaves through the transpiration stream via the xylem. Yang, Feng [61] explore that cation ATPases or ion channel and cation-proton antiport are involved in xylem loading. Nickel is supplied to meristematic parts of the plants by translocation from old to young leaves, buds, fruits, and seeds, via the phloem. This transport is tightly regulated by metal-ligand complexes and proteins that specifically bind Ni [62].

Yield and yield-related parameters of A1 and A2 lines were slightly increased at low nickel while exposure to high nickel dose gradually reduced yield. Seed yield of A1 and A2 lines were high (17.08 and 15.38%) under 50 mg kg^-1^ Ni, respectively. Karagiannidis, Stavropoulos [63] reported that tomato yield increased (2.5%) under Ni treatment. It is well known that Ni triggers the catalytic activity of the urease enzyme [44]. A decline in urease activity seriously affects the amino acids and reduces carbon and nitrogen metabolism [64]. For example, Malavolta and Moraes [65] also documented a high yield in soybean under Ni application. It has been reported that exposure of 25 mg kg^-1^ Ni to the rose of Jamaica elevated fresh and dry biomass. This increment increases the elements like nitrogen, potassium, phosphorus, zinc, and manganese, which had a key role in plant dry matter [66].

The article "Phytoremediation of nickel by quinoa: Morphological and physiological response" was retracted in 2022. Reasons: compromised peer review; a conflict of interest; concerns about the authorship.

## 5. Conclusion

In conclusion, quinoa A2 is a more efficient phytoremediator of Ni-contaminated soils. Substantial reduction in quinoa growth and yield of quinoa lines A7 and A9 were observed with the increase in Ni concentration. Quinoa A2 line showed high translocation of Ni in shoot without showing any adverse effect on growth. This indicates that A2 has the maximum genetic potential for the safe storage of Ni in the shoot. The possible mechanisms involved are better growth, diverse morpho-anatomical features, Ni sequestration with carotenoids and phenolic, metabolic adjustments, and keeping maximum nutrients in plant parts. Importantly Ni concentrations determined in seed samples of all lines were found below the permissible value set (67 mg kg^-1^) by FAO/WHO. This information can be used to design novel breeding strategies such as precise backcrossing of these quinoa germplasm by identifying suitable developmental genes into regionally adapted some other cultivars to improve yield under other low-yielding environments to secure the rising global food demand for cereals. Further, the detailed mechanism of Ni toxicity, sequestration, and compartmentalization using other amendments are needed to be investigated by considering the risk assessment of higher toxic levels.

## Supporting information

S1 Data (XLSX)
